# Down-regulation of miR-10a-5p promotes proliferation and restricts apoptosis via targeting T-box transcription factor 5 in inflamed synoviocytes

**DOI:** 10.1042/BSR20180003

**Published:** 2018-04-13

**Authors:** Nazim Hussain, Wenhua Zhu, Congshan Jiang, Jing Xu, Manman Geng, Xiaoying Wu, Safdar Hussain, Bo Wang, Muhammad Shahid Riaz Rajoka, Yue Li, Juan Tian, Liesu Meng, Shemin Lu

**Affiliations:** 1 Department of Biochemistry and Molecular Biology, School of Basic Medical Sciences, Xi’an Jiaotong University Health Science Center, Xi’an, Shaanxi 710061, China; 2 Key Laboratory of Environment and Genes Related to Diseases (Xi’an Jiaotong University), Ministry of Education, Xi’an, Shaanxi 710061, China; 3 Center for Translational Medicine, the First Affiliated Hospital of Xi’an Jiaotong University, Xi’an, Shaanxi 710061, China; 4 Key Laboratory for Space Science and Biotechnology, School of Life Sciences, Northwestern Polytechnical University, Xi’an, Shaanxi 710072, China; 5 Department of Rheumatology and Immunology, the First Affiliated Hospital of Xi’an Jiaotong University, Xi’an, Shaanxi 710061, China

**Keywords:** apoptosis, cell proliferation, miR-10a-5p, synoviocytes, TBX5

## Abstract

Synoviocytes from rheumatoid arthritis (RA) patients share certain features with tumor cells, such as over proliferation and invasion. Anomalous microRNA (miRNA) expression may participate in the pathogenesis of RA in different ways. The objective of the present study was to observe the role of miR-10a-5p targeting T-box transcription factor 5 (TBX5) gene on synoviocyte proliferation and apoptosis in RA. Human synovial sarcoma cell line, SW982 cells stimulating with interleukin-1β (IL-1β) were transfected with miR-10a-5p mimic and siRNA of TBX5. The real-time quantitative polymerase chain reaction (RT-qPCR) and Western blotting analysis were used to evaluate the expression level of miR-10a-5p and TBX5 in SW982 cells respectively. Further, the proliferation and apoptosis of SW982 cells after treatment were determined by cell counting kit (CCK-8) and flow cytometry analysis respectively. We found that the miR-10a-5p showed down-regulated while TBX5 showed up-regulated expression in synoviocytes after stimulation with IL-1β. The miR-10a-5p mimic treatment showed a decline in cell proliferation while the increased rate of cell apoptosis as compared with control. Moreover, knockdown of TBX5 favored the apoptosis and reduced the cell proliferation as compared with control group. We conclude that down-regulation of miR-10a-5p promotes proliferation and restricts apoptosis via targeting TBX5 in inflamed synoviocytes.

## Introduction

Rheumatoid arthritis (RA) is a chronic inflammatory autoimmune disease of periphery joints. It has affected approximately 0.5–1% of the world population [1]. Discovering the etiology behind RA is significant in formulating treatment and management approaches. It is believed that both genetic and environmental factors contribute their critical roles in the pathophysiology of RA, and approximately 60% of the risk for developing RA comes from genetic factors. The exact cause of RA remains unclear, while it is believed that one of the substantial pathophysiological aspects of RA is a significant increase in the quantity of resident synovial cells, also known as fibroblast-like synoviocytes (FLS) because of their phenotypic appearance and cellular characteristics similarity with mesenchymal originated cells [2]. FLS are unicellular and highly differentiated cells, performing the function of support, nourishment, as well as lubrication to the joint tissue in normal synovium [3]. However, in the case of joint inflammation, FLS behave like tumor cells and become hyperplastic, invasive, and highly migratory cells, and thus contribute a prominent role both in the establishment and the continuation of RA [4,5].

MicroRNAs (miRNAs) are small non-coding RNA molecules with a length of 18–22 nucleotides that negatively and post-transcriptionally regulate the expression of their target genes. MiRNAs are involved in several biological processes such as proliferation, differentiation, apoptosis, development, angiogenesis, and immune response via regulating their target genes [6]. Particularly, there are many studies showing that miRNAs play critical roles in cell proliferation, differentiation, and apoptosis [7–12]. For example, miR-126 has been reported to participate in the proliferation, invasion, migration, and drug resistance [8,9]. MiR-27a is induced by leucine and participates in leucine-induced proliferation promotion of myoblast [10]. MiR-10b and miR-126 were reported to control cell apoptosis, proliferation, migration, and invasion of endometrial cancer and hepatocellular carcinoma via regulation of HOXB3 and Sox2 expression respectively [11,12]. In another study, it has been found that Hcy can induce apoptosis in HCAECs in a dose-dependent manner which caused the up-regulation in the expression level of caspase-3 while down-regulation of miR-30b. In addition, enforced expression of miR-30b inhibited apoptosis Hcy-induced in HCAECs by down-regulating the caspase-3 expression level [13].

Accumulating evidence confirms that anomalous miRNA expression may participate in the pathogenesis of RA in different ways. Thus, it is interesting and important to find out miRNAs regulating FLS inflammation and proliferation as well as apoptosis in arthritis, which would provide valuable targets for therapy of the disease. Recently, we found that down-regulation of miR-10a-5p in synoviocytes contributes to joint inflammation via targeting T-box transcription factor 5 (TBX5) [14]. Decrease in miR-10a-5p and increase in TBX5 could induce the production of proinflammatory cytokines and chemokine, but the role of miR-10a-5p in other aspects of synoviocytes remains poorly understood. In the present study, we intended to explore the role of miR-10a-5p and its target gene TBX5 in apoptosis and proliferation processes of synoviocytes, which would be an important supplement for the function of miR-10a-5p. We consider that this molecular mechanism based on miR-10a-5p function would provide useful clues for the treatment of RA patients.

## Materials and methods

### Cells

Human synovial sarcoma cell line SW982 cells were cultured in Dulbecco’s modified Eagle’s medium (DMEM) supplemented with 10% fetal bovine serum. Cells were incubated at 37°C in a 5% CO_2_ humidified incubator.

### Interleukin-1β (IL-1β) stimulation

The SW982 cells (2 × 10^5^ cells/ml) were cultured into six-well plates until a confluence of cells was reached between 70 and 80%. IL-1β (10 ng/ml) was then added to the plates. The cells were then harvested for RNA and protein extraction at 24 and 48 h after IL-1β stimulation respectively.

### Cell transfection

Before the transfection of SW982 cells, cells were cultured in 12-well or 6-well plates for 24 h. MiRNA control mimic (5′-UUG UAC UAC ACA AAA GUA CUG-3′), miR-10a-5p mimic (5′-UAC CCU GUA GAU CCG AAU UUG UG-3′), siRNA of TBX5 (Si-TBX5) (F: 5′-GGG CAC GGA AAU GAU CAU ATT-3′; R: 5′-UAU GAU CAU UUC CGU GCC CTT-3′), and negative control (si-NC) (F: 5′-UUC UCC GAA CGU GUC ACG UTT-3′; R: 5′-ACG UGA CAC GUU CGG AGA ATT-3′) (Gene Pharma, Shanghai, China) were transfected at a final concentration of 50 nM with Lipofectamine 2000 (Invitrogen, U.S.A.). After 24 and 48 h of transfection, RNA and protein were extracted respectively.

### Real-time quantitative polymerase chain reaction (RT-qPCR)

The cells of SW982 were collected after different treatments. MiR-10a-5p expression level was evaluated by RT-qPCR. Total RNA was extracted from cells using Trizol® Reagent (Invitrogen), quantified by using Nanodrop. A total RNA of 0.45 μg was used in a miRNA-specific stem–loop reverse transcription (RT) reaction for miRNAs, and 2 μg for the RT reaction using oligo d(T) primer. Then cDNA was synthesized by RevertAid™ First Strand cDNA Synthesis Kit (Fermentas). RT-qPCR was performed by iQ5 (Bio-Rad) with SYBR® Premix Ex Taq™ *II* (Takara) for quantification. The relative expression level of miR-10a-5p was normalized by U6 snRNA. All data were analyzed by using 2^−ΔΔ*C*_t_^ (relative quantification) method. The information about genes, primer sequences, and annealing temperatures has been described in Table 1.

**Table 1:** List of primers for RT-qPCR

Gene	Sequences	*T*_a_ (°C)
*miRNA-10a-5p* (RT)	GTCGTATCCAGTGCAGGGTCCGAGGTATTCGCACTGGATACGACCACAAA	–
*miRNA-10a-5p*	F: CGCTACCCTGTAGATCCGAA	60
	R: GTGCAGGGTCCGAGGT	
*U6*	F: CTCGCTTCGGCAGCACA	60
	R: AACGCTTCACGAATTTGCGT	

### Western blotting

Total proteins were extracted from all samples with RIPA lysis buffer and then quantified by using BCA kit (Thermo, U.S.A.). All protein samples with equal amounts of approxiamtely 30 μg were loaded on a 10% SDS denatured polyacrylamide gel (SDS/PAGE) and then transferred to polyvinylidene difluoride membranes (Amersham, Buckinghamshire, U.K.). After 2 h of blocking with 5% fat-free milk, the membranes were then subsequently incubated with the polyclonal anti-TBX5 antibody (1:500, Abcam, USA), or GAPDH (1:10,000, Proteintech, Chicago, U.S.A.) overnight. The membranes were then washed with 1× TBST, and incubated with a horseradish peroxidase-conjugated (HRP-conjugated) secondary antibody for 2 h. Protein expression was evaluated by Supersignal® West Pico kit (Thermo Scientific).

### Cell counting kit-8 (CCK-8)

After transfection with mimic miR-10a-5p or si-TBX5, SW982 cells were cultured in 96-well plates. The CCK-8 (10 μl) (Beyotime Biotechnology, Shanghai, China) was added to wells containing 100 μl of culture medium for 4-h incubation. The optical density (OD) value was obtained at the wavelength of 450 nm by multiskan spectrum (Thermo, U.S.A.). Cell proliferation assay was measured at different time points as indicated.

### Cell apoptosis assay

An apoptosis detection kit (7Sea Pharmatech, China) was used to determine apoptotic cells according to the manufacturer’s instructions. After 48 h of transfection with mimic miR-10a-5p or si-TBX5, SW982 cells were treated with trypsin and collected in 1.5 ml tubes. After washing cells with 1 ml of PBS, 400 μl of Annexin V-FITC binding buffer was added to each tube. The cells were then treated with 5 μl of AnnexinV-FITC at room temperature for 15 min in dark condition. After 15 min cells were then resuspended with 10 μl of PI keeping the tubes in ice up to 5 min. Afterward, flow cytometry was used to analyze cell apoptosis by adding 200 μl of cell suspension into wells of 96-well plate. Cells were analyzed using Guava machine (Millipore, U.S.A.).

### Statistical analyses

All data were presented as mean ± standard error of the mean (SEM), and the statistically significant difference between experimental and control groups was then determined by using Student’s *t*-test. *P*<0.05 was considered to be statistically significant.

## Results

### Expression level of miR-10a-5p is down-regulated in synoviocytes with IL-1β stimulation

Cytokines are considered as principal components with a fundamental role in causing inflammation and articular destruction. IL-1β was used to stimulate human FLS cell line, to mimic the local inflammatory changes in RA. Recently, we have found that miR-10a-5p expression is decreased in the synovium of RA patients as well as in IL-1β stimulated synoviocytes [14]. Here, we used different doses of IL-1β to treat SW982 cells to confirm previous findings. MiR-10a-5p showed gradually down-regulated expression in SW982 cells with the increase in IL-1β concentration, and it was significantly reduced upon 5 and 10 ng/ml IL-1β stimulation (Figure 1A). Thus, SW982 cell line stimulated with IL-1β was used to conduct the further functional experiments.

**Figure 1:** MiR-10a-5p inhibited the proliferation of SW982 cells First, synovial sarcoma cell line (SW982) was stimulated with different doses of IL-1β for 24 h and relative expression level of miR-10a-5p was determined by RT-qPCR (**A**). Expression level of miRNA was normalized by housekeeping genes U6 snRNA. Then, SW982 cells were transfected with miR-10a-5p mimic, and relative expression level of miR-10a-5p was determined by RT-qPCR (**B**). Moreover, miR-10a-5p mimic and NC mimic transfected cells were treated with IL-1β, and cell proliferation was detected at 0, 12, 24, and 48 h by using CCK-8 kit (**C**). Data represent the means ± SEM from three independent experiments; **P<0.01 and ***P<0.001*.*

### Overexpression of miR-10a-5p inhibits the proliferation of synoviocytes

The strategy of overexpressing the miRNAs is useful to understand the regulation of different biological processes including cell proliferation and apoptosis. The expression level of miR-10a-5p was significantly up-regulated up to 90% in SW982 cells after transfection with miR-10a-5p mimic (Figure 1B). Then cell proliferation was determined by using the CCK-8 method, and results showed that there was a significant decrease in miR-10a-5p mimic transfected group compared with NC mimic transfected group (Figure 1C). Our findings suggested that up-regulation of miRNA-10a-5p can resist the proliferation of synoviocytes.

### Overexpression of miR-10a-5p promotes programmed cell death of synoviocytes

On the other hand, miRNAs have pivotal roles in the regulation of cell apoptosis. The results of flow cytometry showed that the percentage of Annexin V-FITC and PI double positive cells was significantly increased in miR-10a-5p mimic transfected group compared with NC group, indicating an increased rate of apoptosis in miR-10a-5p overexpressed synoviocytes (Figure 2A,B). Therefore, we conclude that miR-10a-5p could inhibit cell proliferation but promote synoviocyte apoptosis, besides contributing to inflammation.

**Figure 2:** MiR-10a-5p promoted the apoptosis of SW982 cells SW982 cells were transfected with miR-10a-5p mimic or NC mimic and treated with IL-1β for 24 h, and cell apoptosis was detected by flow cytometer (**A**). Percentage of apoptotic cells was shown in the histogram (**B**). Data represent the means ± SEM from three independent experiments; ***P< 0.001*.*

### Knockdown of TBX5 suppresses proliferation of synoviocytes

We have confirmed that miR-10a-5p targets TBX5 to be involved into joint inflammation, but whether TBX5 also participated in the regulation of cell proliferation and apoptosis remained unclear. TBX5 showed significantly up-regulated expression in SW982 cells after stimulation with IL-1β, which was consistent with previous findings (Figure 3A). Then SW982 cells were transfected with si-TBX5 or si-NC, and Western blotting results showed significant down-regulation in the expression level of TBX5 in si-TBX5 transfected group (Figure 3B). Moreover, with IL-1β stimulation, the cell proliferation rate was significantly reduced in TBX5 knockdown cells, indicating that TBX5 could promote cell proliferation (Figure 3C).

**Figure 3:** Knocking down TBX5 in SW982 cells inhibited cell proliferation SW982 cells were treated with different doses of IL-1β and expression level of TBX5 protein was detected by Western blotting (**A**). GAPDH was used as a housekeeping control. Then, SW982 cells were transfected with Si-TBX5 or si-NC, and the knocking down efficiency was evaluated by detecting TBX5 expression (**B**). Moreover, IL-1β was used to stimulate si-TBX5 or si-NC transfected cells, and cell proliferation was detected at 0, 12, 24, and 48 h by using CCK-8 kit (**C**). Data represent the means ± SEM of three independent experiments; *P<0.05, **P<0.01, ***P<0.001.

### Down-regulation of TBX5 promotes the apoptosis of synoviocytes

In addition, cell apoptosis was also observed under TBX5 down-regulation condition. Flow cytometer results showed that the percentage of Annexin V-FITC and PI double positive cells (apoptotic cells) was significantly increased in si-TBX5 transfected group compared with NC group, indicating an increased rate of apoptosis in synoviocytes with low expression of TBX5 (Figure 4A,B). Summarily, we have proved that TBX5 regulated by miR-10a-5p could promote synoviocyte proliferation and suppress apoptosis, which reveals a new mechanism of miR-10-5p and its target TBX5 in arthritis.

**Figure 4:** TBX5 down-regulation facilitated programmed cell death in SW982 cells SW982 cells were transfected with Si-TBX5 or si-NC and treated with IL-1β for 24 h, and cell apoptosis was detected by flow cytometer (**A**). Percentage of apoptotic cells was shown in the histogram (**B**). Data represent the means ± SEM from three independent experiments; ***P<0.001*.*

## Discussion

RA is an autoimmune chronic inflammatory disorder characterized by a momentous increase in the number of synoviocytes, which results in disproportion between the proliferation and apoptosis of the FLS [15]. They produce cytokines that perpetuate inflammation and MMPs that contribute to the demolition of cartilage in RA. Meanwhile, FLS of RA patients becomes incursive, aggressive, and resistive to apoptosis. Recently, targeting FLS in RA is considered as a strategy for advanced therapies to improve the course of the disease.

A number of studies have proved that unusual expression of miRNAs in disease condition is not by chance but mostly functions in arthritis [16], in which miR-10a-5p is vital one involving in joint inflammation. In our previous study, we found that the level of miR-10a-5p was less in RA synovium than that in osteoarthritis (OA) [14]. Another study also reported that miR-10a expression level was down-regulated in the synovial tissues and FLSs of RA patients [17]. The stimulation of tumor necrosis factor-α (TNF-α) and IL-1β could induce the expression of miR-146a/b and miR-155 in RA synovial fibroblasts remarkably, providing the evidence that miRNAs not only contribute to various aspects of RA pathogenesis, but may also be changed by the inflammatory milieu of resident cells in RA joints [18,19]. The potential role of cytokines in the pathogenesis of RA is a reality and has been revealed after the successful treatment of RA patients with anti-TNF-α antibodies [20]. IL-1β is one of the important and classical proinflammatory cytokines and a strong inducer of chemokines, inflammatory proteins, adhesion molecules, and has the potential to change features of FLS [21]. A number of studies have revealed that miRNAs regulate the expression levels of IL-1β and also IL-1β is involved to control the expression level of miRNAs in RA patients. Our results showed that the expression of miR-10a-5p was down-regulated after stimulation with IL-1β, although the mechanism by which the expression of miR-10a-5p is regulated is not yet clear.

In the present study, for better and more comprehensive understanding and explanation of RA-related mechanism of miR-10a-5p, we tried to investigate its potential function in proliferation and apoptosis, although we have revealed the role of miR-10a-5p in controlling inflammatory cytokine production in arthritis. Mounting evidence has reported that miR-10a regulates cell proliferation, migration, and invasion, and hence plays essential roles in a variety of cancers, for example, extrahepatic cholangiocarcinoma, prostate, colon cancer, esophageal squamous cell carcinoma, and head and neck squamous cell carcinoma [22–25]. Reduced expression of miR-10a triggers the activation of nuclear factor-κB (NF-κB) signaling pathway and promotes the proinflammatory factors [26], which results in increased cell proliferation, migration, invasiveness or angiogenesis, decreased apoptosis or dedifferentiation. However, the role in FLS of RA remained poorly understood. We found that miR-10a-5p can promote proliferation and inhibits apoptosis in inflamed synoviocytes, suggesting that low expression levels of miR-10a-5p during the pathogenesis of RA could have momentous effects on synovial cell proliferation and apoptosis processes.

In our previous study, TBX5 was confirmed as a target gene of miR-10a-5p [14]. TBX5 is a member of T-box transcription factor family; in which each candidate shares a common T-box DNA-binding domain in their sequences. It has been recognized as a well-known transcription factor which plays an important role in tissue development, cancer, and a number of other biological activities. However, little was known about the role of TBX5 in arthritis before. Recently, it was reported that TBX5 was less methylated in the synovium and FLS of RA patients than in OA samples [27]. We found that miR-10a-5p targeting TBX5 play their role in joint inflammation.

In the present study as successive work, we found that down-regulated expression of TBX5 caused the reduction in proliferation, while increased the apoptosis rate of synoviocytes. Thus, miR-10a-5p might modulate cell apoptosis, the proliferation of synoviocytes via targeting TBX5, which is an important supplementary mechanism to miR-10a-5p in arthritis. Interestingly, TBX5 was reported as a tumor suppressor and recognized as a biomarker for colon cancer [28]. In addition, the TBX5 actions on transcriptional regulation contributed to induction of apoptosis and inhibition of cell proliferation [29,30]. It indicated that TBX5 might play different roles in modulating cell proliferation and apoptosis when cells were under different pathological and physiological conditions.

Currently, miRNAs are considered as a new class of potential therapeutic targets, while the process of their biosynthesis, maturation, and regulation can be influenced by using oligonucleotides [31]. Several studies on miRNA-based treatment have been performed in animal models [32]. Hence, miRNA-based therapy is a brilliant method of treating RA, and our findings might present a potential therapeutic target, miR-10a-5p, for the treatment of RA patients. Though, limitations persist in the present study. TBX5 is a transcription factor, and its target genes participate not only in apoptosis, proliferation, migration, and invasion but also in some other functions. The regulatory mechanism of the miR-10a-5p-TBX5 will be a target of further investigation in our future study.

## Abbreviations

FLS: fibroblast-like synoviocytes
IL-1β: interleukin-1β
miRNA: microRNA
NF-κB: nuclear factor-κB
OA: osteoarthritis
RA: rheumatoid arthritis
RT-qPCR: real-time quantitative polymerase chain reaction
TBX5: T-box transcription factor 5
TNF-α: tumor necrosis factor-α
